The article "Mitophagy Impairment Aggravates Cisplatin-Induced Ototoxicity" was published in 2021. Journal: Biomed Res Int.

# Mitophagy Impairment Aggravates Cisplatin-Induced Ototoxicity

**DOI:** 10.1155/2021/5590973

**Published:** 2021-05-20

**Authors:** Sung Il Cho, Eu-Ri Jo, Hansoo Song

**Affiliations:** ^1^Department of Otolaryngology-Head and Neck Surgery, Chosun University College of Medicine, Gwangju, Republic of Korea; ^2^Department of Occupational & Environmental Medicine, Chosun University College of Medicine, Gwangju, Republic of Korea

## Abstract

Cisplatin is an efficacious anticancer agent, but its use is limited by ototoxicity and resultant irreversible sensorineural hearing loss. Cisplatin ototoxicity is associated with cochlear cell oxidative stress and mitochondrial damage. However, mitophagy is vital for maintaining mitochondrial quality and cellular metabolism. Accordingly, we investigated the role of mitophagy in regulating cisplatin-induced ototoxicity using the auditory cell line HEI-OC1. In this study, HEI-OC1 cells were treated with either cisplatin alone (10 *μ*M, 0, 8, 16, and 24 h); cisplatin (10 *μ*M, 24 h) post transfection with small-interfering (si)RNAs targeting mitophagy-associated mRNAs; cisplatin (10 *μ*M, 24 h) succeeding pretreatment with the mitophagy suppressor, 3-methyladenine (3-MA; 5 or 10 mM, 6 h); or cisplatin (30 *μ*M, 24 h) following pretreatment with the mitophagy promoter, carbonyl cyanide m-chlorophenylhydrazone (CCCP; 1 or 2 *μ*M, 2 h). The viability of cells, expression of mitophagy marker, and mitochondrial functions were then assessed in these cells. Cell viability was determined by a water-soluble tetrazolium assay; expression of mitophagy-associated proteins *PINK1*, *Parkin*, *BNIP3*, *FUNDC1*, p62, and LC3B was analyzed by Western blotting, mitochondrial membrane potential by flow cytometry, intracellular ATP by spectrophotometry, and mitochondrial degradation by dual staining for mitochondria and autophagosomes or lysosomes. Our results showed that cisplatin gradually reduced the viable cell number over time, induced mitochondrial depolarization, decreased intracellular ATP concentration, and enhanced the expression of *PINK1*, *Parkin*, *BNIP3*, p62, and LC3B. In addition, *Parkin* and *BNIP3* knockdown accelerated cisplatin-induced loss of cell viability, mitochondrial membrane potential, mitophagosome/lysosome formation, and reduction in intracellular ATP production. Pretreatment with 3-MA aggravated the cisplatin-induced cytotoxicity, while that with CCCP reversed this effect. Overall, our findings indicate that mitophagy protects HEI-OC1 cells against cisplatin-induced cell death. Consequently, we strongly believe that targeted promotion of mitophagy may confer protection against cisplatin-induced ototoxicity.

The article "Mitophagy Impairment Aggravates Cisplatin-Induced Ototoxicity" was published in 2021. Journal: Biomed Res Int.

## 1. Introduction

Cisplatin (cis-diamminedichloroplatinum II) is the most widely used chemotherapeutic agent for both pediatric and adult cancer patients owing to its broad-spectrum antitumor efficacy [1]. However, cisplatin chemotherapy causes bilateral, irreversible, and progressive hearing loss in 40%–80% of patients [2, 3]. This hearing loss results at least in part from excessive reactive oxygen species (ROS) generation in cochlear cells, leading to mitochondrial damage, metabolic disruption, and cell death [3]. Mitochondria generate adenosine triphosphate (ATP) required for most cellular activities via the tricarboxylic acid cycle and oxidative phosphorylation (OXPHOS). Moreover, mitochondria control redox homeostasis, Ca^2+^ signaling, and iron metabolism [4]. Dysfunctional mitochondria release cytochrome c and proapoptotic factors into the cytoplasm that trigger apoptosis [5]. To prevent apoptosis and maintain cellular energy, the mitochondrial pool is subject to constant turnover through biogenesis and mitophagy, which is a mitochondria-specific form of autophagy that selectively degrades damaged mitochondria via the autophagosome-lysosome pathway. Undeniably, the maintenance of mitochondrial turnover is critical for long-term cellular fitness [6].

Alternatively, impaired mitophagy results in the accumulation of dysfunctional mitochondria, leading to inadequate ATP production, augmented ROS production, and ultimate cell death. In addition, impaired mitophagy is associated with aging, inflammation, neurodegenerative diseases, and cancer [7]. To examine if impaired or insufficient mitophagy contributes to cisplatin-induced ototoxicity, we compared the viability and metabolic capacity of an auditory cell line that was treated with cisplatin under the conditions of enhanced or inhibited mitophagy.

## 2. Materials and Methods

### 2.1. Cell Culture and Cell Viability Assay

The House Ear Institute-Organ of Corti 1 (HEI-OC1) cell line was used as an in vitro model to investigate the mechanisms of ototoxicity as these cells express molecular markers characteristic of the organ of Corti as well as supporting cells [8]. The cells were cultured in Dulbecco's modified Eagle medium (WelGENE Inc., Daegu, South Korea) supplemented with 10% fetal bovine serum (Lonza, Walkersville, MD, USA) at 33°C under an atmosphere of 5% CO_2_ in a humidified incubator. To determine the effect of cisplatin treatment on cell viability and the influence of mitophagy, HEI-OC1 (8 × 10^4^) cells were seeded per well in 24-well plates for 24 h. They were then subjected to treatment with 10 *μ*M cisplatin alone for 0, 8, 16, and 24 h; 10 *μ*M cisplatin for 24 h post transfection with siRNAs targeting mitophagy-associated mRNAs for 48 h; 10 *μ*M cisplatin for 24 h following a 6 h pretreatment with the mitophagy suppressor, 3-methyladenine (3-MA; Sigma, St. Louis, MO, USA); or 30 *μ*M cisplatin for 24 h post a 2 h pretreatment with the mitophagy promoter carbonyl cyanide m-chlorophenylhydrazone (CCCP; Sigma). Cell viability was determined using the water-soluble tetrazolium salt- (WST-) based EZ-Cytox cell viability assay kit (Daeil Lab Service Co., Seoul, South Korea). After the indicated treatments, the cells were incubated with 50 *μ*L WST solution in 450 *μ*L culture media for 2 h at 33°C. The WST metabolic product generated by viable cells was then measured by the absorbance at 450 nm using a spectrophotometer (BioTek, Winooski, VT, USA).

The article "Mitophagy Impairment Aggravates Cisplatin-Induced Ototoxicity" was published in 2021. Journal: Biomed Res Int.

### 2.2. Transfection of siRNAs

HEI-OC1 (2 × 10^5^) cells were seeded per well in 6-well plates for 24 h and then transfected with si-Control, si-*Parkin*, or si-*BNIP3* (Santa Cruz Biotechnology, Dallas, TX, USA) for 48 h using the Lipofectamine® RNAiMAX reagent (Invitrogen, Carlsbad, CA, USA) according to the manufacturer's protocol. Subsequently, the transfected cells were treated with cisplatin as indicated.

### 2.3. Western Blot Analysis

To extract mitochondrial proteins, HEI-OC1 cells post indicated treatments were harvested, washed with phosphate-buffered saline (PBS), suspended in cytosol extraction buffer (75 mm NaCl, 8 mM Na_2_HPO_4_, 1 mM NaH_2_PO_4_, 250 mM sucrose, 1 mM EDTA, and 350 *μ*g/mL digitonin) for 5 min on ice, and centrifuged at 13000 rpm for 20 min at 4°C. The supernatant (cytosolic fraction) was discarded, and the pellet containing isolated mitochondria was washed with PBS, centrifuged as described earlier, resuspended in lysis buffer for 10 min on ice, and centrifuged at 13000 rpm for 10 min at 4°C. The supernatant was used as the mitochondrial protein fraction. Protein samples were boiled in SDS-PAGE sample buffer, separated using 12% polyacrylamide gels, and transferred onto PVDF membranes (Millipore Corp, Danvers, MA, USA). The membranes were blocked with 5% skim milk in TBS-T (20 mM Tris-HCl, 137 mM NaCl, pH 7.5, and 0.1% Tween-20) for 1 h at room temperature and then incubated with primary antibodies against *PINK1*, *Parkin*, *BNIP3* (Thermo Fisher Scientific, Waltham, MA, USA), *FUNDC1*, p62, LC3B, and COX IV (Cell Signaling Technology, Danvers, MA, USA). Blotted membranes were washed thrice with TBS-T (10 min/wash) and incubated with sheep anti-mouse and donkey anti-rabbit IgGs conjugated to X (Jackson ImmunoResearch, West Grove, PA, USA). The membranes were washed three times with TBS-T (10 min/wash), and protein band densities were quantified using a Western blot detection system (Millipore) and image analyzer (Vilber, Collégien, France).

The article "Mitophagy Impairment Aggravates Cisplatin-Induced Ototoxicity" was published in 2021. Journal: Biomed Res Int.

### 2.4. Immunofluorescence Analysis

HEI-OC1 cells were seeded onto sterile 12 mm glass coverslips in 6-well plates and subjected to indicated treatments. Post treatments, the cells were stained with 200 nM MitoTracker® Red CMXRos (Thermo Fisher Scientific, Waltham, MA, USA) for 20 min in Opti-MEM® Reduced Serum Medium (Thermo Fisher Scientific) for staining mitochondria. They were then washed twice with PBS and fixed using 100% methanol for 15 min. Subsequently, the fixed cells were washed twice with PBS, blocked in 1% BSA solution, and incubated with anti-LC3B (Cell Signaling Technology) and anti-LAMP1 (Santa Cruz Biotechnology) antibodies overnight at 4°C. The cells were then washed twice with PBS and incubated with FITC-conjugated chicken anti-mouse and Alexa Fluor 488 conjugated anti-goat antibodies (Invitrogen) for 2 h. After washing in PBS, the labeled cells were mounted on slides using Fluorescent Mounting Medium with DAPI (GBI Labs, Bothell, WA, USA). Immunofluorescence was detected by confocal microscopy (Carl Zeiss, Oberkochen, Germany) and ZEN imaging software ZEN (Carl Zeiss). Colocalization coefficients were quantified using NIH-ImageJ software (National Institutes of Health, Bethesda, MD, USA).

### 2.5. Measurement of Mitochondrial Membrane Potential

Mitochondrial membrane potential was estimated using MitoTracker® Red CMXRos (Thermo Fisher Scientific, Waltham, MA, USA). Briefly, the HEI-OC1 cells were treated as indicated in 6-well plates and stained with 200 nM MitoTracker® Red CMXRos for 20 min in Opti-MEM® Reduced Serum Medium (Thermo Fisher Scientific). After staining, the cells were harvested, washed twice with PBS, and centrifuged to obtain the cell pellet. The cellular fluorescence intensity was measured by flow cytometry (BD Biosciences, San Diego, CA, USA) and analyzed using Cell Quest software (BD Biosciences).

### 2.6. Measurement of Intracellular ATP Content

Intracellular ATP was measured using an ATP Assay Kit (BioVision, Milpitas, CA, USA) following the manufacturer's protocol. The absorbance values of samples and standards were measured at 570 nm using a spectrophotometer (BioTek), and ATP concentrations were determined based on a standard curve. Values are expressed as nmol/*μ*L (per 10^5^ cells) relative to si-Control cultures.

### 2.7. Statistical Analysis

All results were analyzed using SPSS 24.0 (IBM Corp., Armonk, NY, USA). Cell viability, mitophagy-associated protein expression, mitochondrial membrane potential, and ATP content were compared between the treatment groups using Student's *t*-test. *p* < 0.05 (two-tailed) was considered statistically significant for all tests.

The article "Mitophagy Impairment Aggravates Cisplatin-Induced Ototoxicity" was published in 2021. Journal: Biomed Res Int.

## 3. Results

### 3.1. Cisplatin Reduces the HEI-OC1 Cell Viability and Increases the Expression of Mitophagy-Associated Proteins

To assess the effect of cisplatin on the viability and mitophagy of HEI-OC1 cells, the cells were subject to the assessment of cell viability and mitophagy-related marker expression, post cisplatin treatment. Our results revealed that cisplatin treatment (10 *μ*M) induces a time-dependent decline in the number of viable HEI-OC1 cells as compared to the untreated controls (98.4% ± 0.8% vs. untreated controls after 8 h, 92.8% ± 0.6% after 16 h, and 85.3% ± 1.5% after 24 h) (Figure 1(a)). In contrast, relative expression levels of the mitophagy-associated proteins including *PINK1*, *Parkin*, and *BNIP3* as well as the autophagosome markers LC3B and p62 evidently increased in the mitochondrial protein extracts upon cisplatin exposure in a time-dependent manner (*n* = 5 independent experiments, *p* < 0.01, Figures 1(b) and 1(c)). However, there was no significant change in FUNDC1 levels post cisplatin exposure. These results indicate that exposure to cisplatin accelerates mitophagy in HEI-OC1 cells.

### 3.2. Knockdown of *Parkin* and *BNIP3* Aggravates the Cisplatin-Induced Decline in HEI-OC1 Cell Viability

The *PINK1*/*Parkin* and *BNIP3*/*Nix* pathways control the degradation of damaged mitochondria via mitophagy. Transfection of HEI-OC1 cells with siRNAs targeting *Parkin* and *BNIP3* mRNAs significantly accelerates the decrease in cisplatin exposure-induced cell viability (*n* = 5 independent experiments, *p* < 0.01, Figure 2(a)). Further, the expression levels of *PINK1* and LC3B as well as *Parkin* and *BNIP3* were markedly reduced post siRNA-mediated knockdown of *Parkin* and *BNIP3* (*n* = 5 independent experiments, *p* < 0.05, Figures 2(b) and 2(c)), suggesting that mitophagy was strongly inhibited. Mitophagy is a degradative process mediated by the formation of mitophagosomes containing dysfunctional mitochondria that are subsequently fused with lysosomes. The generation of mitophagosomes and mitophagolysosomes was investigated by analyzing colocalization of the mitochondrial stain MitoTracker with the autophagosome marker LC3B and the lysosomal marker LAMP1, respectively. Knockdown of *Parkin* and *BNIP3* mRNAs in HEI-OC1 cells significantly reduces the formation of mitophagosomes and mitophagolysosomes (*n* = 5 independent experiments, *p* < 0.01, Figures 3(a) and 3(b)), strongly suggesting that disruption of mitophagy aggravates the cisplatin-induced cytotoxicity in HEI-OC1 cells.

### 3.3. Knockdown of *Parkin* and *BNIP3* Exacerbates Cisplatin-Induced Mitochondrial Dysfunction in HEI-OC1 Cells

To investigate if *Parkin* and *BNIP3* mRNA knockdown can indeed lead to the accumulation of dysfunctional mitochondria via suppression of mitophagy, we measured the mitochondrial membrane potential and intracellular ATP content in HEI-OC1 cells transfected with respective siRNAs. Our results revealed that mitochondrial depolarization increases following cisplatin treatment of HEI-OC1 cells and was further impaired upon knockdown of *Parkin* and *BNIP3* (*n* = 5 independent experiments, *p* < 0.01, Figures 4(a)and 4(b)). In addition, the knockdown of *Parkin* and *BNIP3* also enhances the cisplatin-induced reduction in cellular ATP concentration (*n* = 5, *p* < 0.01, Figure 4(c)), consistent with increased accumulation of damaged mitochondria in HEI-OC1 cells.

The article "Mitophagy Impairment Aggravates Cisplatin-Induced Ototoxicity" was published in 2021. Journal: Biomed Res Int.

### 3.4. Chemical Inhibition of Mitophagy Enhances Cisplatin Cytotoxicity in HEI-OC1 Cells

To further validate the notion that mitophagy impairment accelerates cisplatin-induced cytotoxicity, we compared the viable cell numbers between cells treated with cisplatin alone to cultures first pretreated with 3-MA, a class III phosphatidylinositol 3-kinase inhibitor and a mitophagy suppressor (5 and 10 mM), before cisplatin exposure. Consistent with insufficient mitophagy as a contributor to cisplatin-induced ototoxicity, our results indicate that 3-MA pretreatment reduces the survival of HEI-OC1 cells post cisplatin treatment as compared to the treatment with cisplatin alone (*n* = 5 independent experiments, *p* < 0.01, Figure 5(a)) in a dose-dependent manner. The expression levels of *PINK1*, *Parkin*, *BNIP3*, and LC3B are also dose-dependently reduced by 3-MA pretreatment prior to cisplatin exposure as compared to those by cisplatin exposure alone (*n* = 5 independent experiments, *p* < 0.01, Figures 5(b) and 5(c)). Thus, our findings suggest that inhibition of mitophagy aggravates the cisplatin-induced damage to HEI-OC1 cells.

### 3.5. Enhanced Mitophagy Reverses the Cisplatin-Induced Cytotoxicity in HEI-OC1 Cells

To determine whether mitophagy activation inhibits cisplatin-induced cytotoxicity, we compared cell viability between HEI-OC1 cells treated with cisplatin alone and cells pretreated with CCCP (1 and 2 *μ*M, 2 h) prior to cisplatin exposure. Our results showed that CCCP pretreatment significantly enhances the survival of HEI-OC1 cells (*n* = 5 independent experiments, *p* < 0.05, Figure 6(a)). Furthermore, the expression levels of *PINK1*, *Parkin*, *BNIP3*, and LC3B were additionally augmented by CCCP pretreatment prior to cisplatin exposure as compared to those by cisplatin exposure alone (*n* = 5 independent experiments, *p* < 0.05, Figures 6(b) and 6(c)). These findings strongly suggest that the cytoprotective effects of CCCP on HEI-OC1 cells exposed to cisplatin are mediated by accelerated mitophagy.

The article "Mitophagy Impairment Aggravates Cisplatin-Induced Ototoxicity" was published in 2021. Journal: Biomed Res Int.

## 4. Discussion

Mitochondria transform nutrients and oxygen into ATP via OXPHOS to power cellular proliferation, motility, signal transduction, and ionic redistribution among a countless number of other processes. However, OXPHOS is also a major generator of ROS, especially under stressful conditions [9]. Moreover, ROS generation by stressed or dysfunctional mitochondria perpetuates further ROS generation by damaging mitochondrial DNA (mtDNA) and proteins, including the electron transporters and membrane pumps mediating OXPHOS. When this functional impairment reaches a threshold, mitochondrial membrane potential is lost, resulting in cell death [10]. Cisplatin exposure increases intracellular ROS production and depletes antioxidant enzymes in cochlear cells, suggesting that oxidative stress contributes to cisplatin-induced ototoxicity [9]. Cisplatin is associated with endoplasmic reticulum stress in addition to the damage of mitochondrial function [11]. Inhibition of endoplasmic reticulum stress has been shown to restore mitochondrial function [12]. Though various interventions, including the usage of small molecule compounds and targeted drug delivery systems, have been reported to reduce the ototoxicity of cisplatin, none of them has been granted FDA approval, and hence, further research is essential [13, 14]. Here, we demonstrate that promotion of mitophagy can alleviate the cisplatin-induced ototoxicity, potentially enhancing the tolerability and efficacy of cisplatin treatment regimens.

Mitophagy maintains cellular metabolism and redox balance by selectively removing superfluous or damaged mitochondria and enabling biosynthesis of new mitochondria [15], thereby conferring cytoprotection under certain conditions [16, 17]. Mitophagy is activated by depolarization of the mitochondrial membrane [18]. In the present study, expression levels of the mitophagy-associated proteins such as *PINK1*, *Parkin*, and *BNIP3* were increased in an auditory cell line post cisplatin exposure. These results indicate the activation of a compensatory protective mechanism under chemical stress. This notion was further validated upon the knockdown of *Parkin* and *BNIP3* that resulted in enhanced cisplatin-induced mitochondrial dysfunction and cytotoxicity in HEI-OC1 cells.

The *PINK1*/*Parkin* pathway is the most extensively investigated mechanism of mitophagy regulation. Both the import and degradation of *PINK1* are reportedly blocked following damage to the mitochondrial membrane potential. The resultant upregulation of *PINK1* causes *Parkin* to bind depolarized mitochondria and translocate into the matrix, where it promotes ubiquitination of mitochondrial proteins and triggers mitophagic degradation [19]. Alternatively, *BNIP3* acts as a key regulator of *Parkin*-independent mitophagy by binding to LC3B on autophagosomes and promoting engulfment of damaged mitochondria [20, 21]. Previous studies have reported that *PINK1*/*Parkin*-mediated mitophagy protects against cisplatin-induced neurotoxicity and nephrotoxicity [22, 23]. Thus, the current results provide further validation to a widespread cellular protective mechanism involving mitophagy.

The article "Mitophagy Impairment Aggravates Cisplatin-Induced Ototoxicity" was published in 2021. Journal: Biomed Res Int.

Whether mitophagy is protective or deleterious to cell survival depends on physiological and pathological context [24]. Under stress, upregulation of mitophagy serves to remove damaged mitochondria and prevent apoptosis. However, this pathway may become overwhelmed by prolonged stress, resulting in cell death [25]. Indeed, the cytotoxic effect of cisplatin progresses slowly over time. 3-MA inhibits autophagy and mitophagy by blocking type III phosphatidylinositol 3 kinases and downstream autophagosome formation [26]. In the current study, inhibition of mitophagy by 3-MA pretreatment aggravated the cisplatin-induced cytotoxicity, consistent with the notion that HEI-OC1 cells are unable to sustain sufficient mitophagy upon cisplatin exposure. Conversely, an activator of mitophagy, the mitochondrial membrane depolarizing agent CCCP [27], actually decreases the cisplatin-induced cytotoxicity which corroborates a previous report suggesting that autophagy suppresses ROS accumulation and oxidative stress in hair cells, thereby preventing cell death [28, 29]. Induction of mitophagy mitigates aging-induced cardiovascular damages [30] in addition to promoting hair cell senescence and aggravating age-related hearing loss [31]. Mitophagy could also lead to the failure of activation of apoptosis and induce resistance of cancer cells to chemotherapeutic treatment [32].

The present study shows that cisplatin exposure induces mitophagy in auditory cells. Knockdown of mitophagy-regulating proteins or inhibition of mitophagy further enhances the severity of cisplatin-induced cytotoxicity. Thus, our results indicate that mitophagy might have a cytoprotective role in cisplatin-induced ototoxicity.

## 5. Conclusion

Cisplatin reduces the viability of auditory cells, an effect that is prevented upon augmenting mitophagy. Thus, promotion of mitophagy may help preserve auditory function in cancer patients receiving cisplatin therapy.

## Figures and Tables

**Figure 1:** Cisplatin reduces the HEI-OC1 cell viability and upregulates mitophagy-associated proteins. HEI-OC1 cells were treated with 10 *μ*M cisplatin for 0 (control), 8, 16, and 24 h. (a) Cell survival decreasing with cisplatin exposure in a time-dependent manner. (b, c) Cisplatin exposure increasing the expression of mitophagy-associated proteins. (b) Representative immunoblots of *PINK1*, *Parkin*, *BNIP3*, *FUNDC1*, p62, LC3B, and COX IV (loading control) from cell lysates harvested after the indicated cisplatin treatment time. (c) Mean changes in the expression of *PINK1*, *Parkin*, *BNIP3*, *FUNDC1*, p62, and LC3B relative to that of COX IV using densitometry analyses. Data are presented as the mean ± standard error of the mean (S.E.M.) of five independent experiments. ^∗^*p* < 0.05; ^∗∗^*p* < 0.01.

The article "Mitophagy Impairment Aggravates Cisplatin-Induced Ototoxicity" was published in 2021. Journal: Biomed Res Int.

**Figure 2:** Knockdown of *Parkin* and *BNIP3* enhances the reduction in HEI-OC1 cell viability following cisplatin (CP) treatment and reduces the expression of mitophagy-associated proteins. (a) The survival rates of HEI-OC1 cells in the si-*Parkin* and si-*BNIP3* transfected groups relative to that in si-Control transfected and cisplatin alone treatment groups. (b) Representative immunoblots of cell lysates harvested after the indicated treatments showing *PINK1*, *Parkin*, *BNIP3*, LC3B, and COX IV (loading control) expression. (c) Relative expression levels of *PINK1*, *Parkin*, *BNIP3*, and LC3B were increased post cisplatin treatment alone but significantly downregulated upon *Parkin* and *BNIP3* siRNA transfection prior to cisplatin treatment. Data presented as the mean ± S.E.M. of five independent experiments. ^∗^*p* < 0.05; ^∗∗^*p* < 0.01.

**Figure 3:** Cisplatin (CP) enhances the rate of mitophagy in HEI-OC1 cells while the knockdown of *Parkin* and *BNIP3* expression reverses this effect. Mitophagosomes and mitophagolysosomes were detected by colocalization (yellow puncta) of LC3B (green) with MitoTracker (red) (a, upper), and LAMP1 (green) with MitoTracker (red) (b, upper), respectively. The area of overlap in HEI-OC1 cells transfected with si-Control was enhanced by cisplatin treatment (10 *μ*M, 24 h), while colocalization areas were significantly reduced in cells transfected with *Parkin* and *BNIP3* siRNAs prior to cisplatin treatment. Data are expressed as the mean ± S.E.M. of five independent experiments. ^∗∗^*p* < 0.01.

**Figure 4:** Knockdown of *Parkin* and *BNIP3* enhances cisplatin- (CP-) induced mitochondrial dysfunction. HEI-OC1 cells were transfected with the indicated siRNAs followed by treatment with cisplatin (10 *μ*M, 24 h). (a) Mitochondrial membrane potential was examined by flow cytometry. (b) Mitochondrial depolarization was significantly greater in cisplatin-treated HEI-OC1 cells transfected with *Parkin* and *BNIP3* siRNAs as compared to cisplatin-treated cells transfected with si-Control. (c) Knockdown of *Parkin* and *BNIP3* impairs the cisplatin-induced reduction of intracellular ATP. Data are presented as the mean ± S.E.M. of five independent experiments. ^∗∗^*p* < 0.01.

The article "Mitophagy Impairment Aggravates Cisplatin-Induced Ototoxicity" was published in 2021. Journal: Biomed Res Int.

**Figure 5:** Chemical inhibition of cisplatin (CP) augmented mitophagy induces cytotoxicity and suppresses the expression of mitophagy-associated proteins. (a) The survival of cisplatin-treated HEI-OC1 cells was significantly reduced by pretreatment with the mitophagy suppressor 3-MA. (b, c) Pretreatment with 3-MA downregulates the expression of *PINK1*, *Parkin*, *BNIP3*, and LC3B in a dose-dependent manner. Data are presented as the mean ± S.E.M. of five independent experiments. 3-MA: 3-methyladenine; ^∗∗^*p* < 0.01.

**Figure 6:** Chemical facilitation of mitophagy protects HEI-OC1 cells from cisplatin- (CP-) induced cytotoxicity and enhances the expression of mitophagy-related proteins. (a) Pretreatment with CCCP prior to cisplatin enhances the survival of HEI-OC1 cells as compared to cisplatin treatment alone. (b, c) CCCP pretreatment upregulates the expression of *PINK1*, *BNIP3*, and LC3B. Data are presented as the mean ± S.E.M. of five independent experiments. CCCP: carbonyl cyanide m-chlorophenylhydrazone; ^∗^*p* < 0.05; ^∗∗^*p* < 0.01.

## Data Availability

Data are available from the corresponding author on request.
